The article "Blockchain-Based Deep Learning to Process IoT Data Acquisition in Cognitive Data" was retracted in 2023. Reasons: signs of a paper mill; compromised peer review; unreliable results or conclusions.

# Blockchain-Based Deep Learning to Process IoT Data Acquisition in Cognitive Data

**DOI:** 10.1155/2022/5038851

**Published:** 2022-02-11

**Authors:** S. Hannah, A. J. Deepa, Varghese S. Chooralil, S. BrillySangeetha, N. Yuvaraj, R. Arshath Raja, C. Suresh, Rahul Vignesh, YasirAbdullahR, K. Srihari, Assefa Alene

**Affiliations:** ^1^Department of Computer, Science and Engineering, Anna University, India; ^2^Department of Computer Science and Engineering, Ponjesly College of Engineering, India; ^3^Department of Computer Science and Engineering, Rajagiri School of Engineering & Technology, India; ^4^Department of Computer Science and Engineering, IES College of Engineering, India; ^5^Research and Development, ICT Academy, IIT Madras Research Park, India; ^6^CSE, Sri Ranganathar Institute of Engineering and Technology, Coimbatore, India; ^7^CSE, Dhanalakshmi Srinivasan College of Engineering, Coimbatore, India; ^8^Department of Computer Science and Engineering, Sri Krishna College of Engineering and Technology, India; ^9^Department of Computer Science and Engineering, SNS College of Technology, India; ^10^Department of Chemical Engineering, College of Biological and Chemical Engineering, Addis Ababa Science and Technology University, Ethiopia

## Abstract

Remote health monitoring can help prevent disease at the earlier stages. The Internet of Things (IoT) concepts have recently advanced, enabling omnipresent monitoring. Easily accessible biomarkers for neurodegenerative disorders, namely, Alzheimer's disease (AD) are needed urgently to assist the diagnoses at its early stages. Due to the severe situations, these systems demand high-quality qualities including availability and accuracy. Deep learning algorithms are promising in such health applications when a large amount of data is available. These solutions are ideal for a distributed blockchain-based IoT system. A good Internet connection is critical to the speed of these system responses. Due to their limited processing capabilities, smart gateway devices cannot implement deep learning algorithms. In this paper, we investigate the use of blockchain-based deep neural networks for higher speed and delivery of healthcare data in a healthcare management system. The study exhibits a real-time health monitoring for classification and assesses the response time and accuracy. The deep learning model classifies the brain diseases as benign or malignant. The study takes into account three different classes to predict the brain disease as benign or malignant that includes AD, mild cognitive impairment, and normal cognitive level. The study involves a series of processing where most of the data are utilized for training these classifiers and ensemble model with a metaclassifier classifying the resultant class. The simulation is conducted to test the efficacy of the model over that of the OASIS-3 dataset, which is a longitudinal neuroimaging, cognitive, clinical, and biomarker dataset for normal aging and AD, and it is further trained and tested on the UDS dataset from ADNI. The results show that the proposed method accurately (98%) responds to the query with high speed retrieval of classified results with an increased training accuracy of 0.539 and testing accuracy of 0.559.

The article "Blockchain-Based Deep Learning to Process IoT Data Acquisition in Cognitive Data" was retracted in 2023. Reasons: signs of a paper mill; compromised peer review; unreliable results or conclusions.

## 1. Introduction

Modern life is being transformed by big data and machine learning, from entertainment to commerce to healthcare. Netflix, Amazon, and Google all know what movies and series people want to watch, what things they like to buy, and what symptoms and ailments they are searching for. All of these data may be used to create extremely complete personal profiles, which can be used for behavioural understanding and marketing, as well as to predict healthcare trends. According to several experts, artificial intelligence (AI) has the potential to revolutionise the healthcare industry, from diagnostics to treatment. An overwhelming amount of evidence suggests that AI algorithms can already perform better than humans in a wide range of activities, such as the analysis of medical pictures and the correlation of illness symptomatology and biomarkers from electronic medical records (EMRs) [1].

Medical professionals, particularly doctors, are in short supply in many nations due to the rising demand for healthcare services. It is not just consumers who are demanding better service and better outcomes from healthcare providers; they are also demanding it from healthcare providers themselves [2]. Using health tracking applications and search platforms, as well as the advancements in wireless technology and cellphones, on-demand healthcare services can now be offered at any time and from any location. Underserved regions and areas without specialists can benefit from these services, which help cut expenses while also preventing the spread of infectious diseases in the clinic. Even in undeveloped countries where the healthcare system is expanding, telehealth technology can be used to satisfy present needs [3]. Although the concept is clear, independent validation is still required to show the safety and efficacy of these treatments for patients.

It is becoming clear that an artificial intelligence- (AI-) powered tool [4–10] will play an important role in the development of next-generation healthcare technology. AI is widely regarded as being capable of improving any aspect of healthcare delivery and operation. AI is gaining traction in the healthcare industry because of its potential to save money.

The article "Blockchain-Based Deep Learning to Process IoT Data Acquisition in Cognitive Data" was retracted in 2023. Reasons: signs of a paper mill; compromised peer review; unreliable results or conclusions.

Alzheimer's disease (AD) is a multifactorial neurodegenerative disorder that affects the central nervous system. It is the most prevalent kind of dementia and is characterised by severe neuronal and synaptic loss. According to a recent study, AD has a high prevalence, with an estimated 40 million sufferers globally. Mild cognitive impairment (MCI) has traditionally been seen as a transitional stage between normal aging and the start of AD. As a result, AD and MCI, the transitional stage between healthy aging and dementia, which is frequently characterised by mild cognitive abnormalities but generally intact activities of daily living, have piqued the interest of researchers.

Changing the healthcare strategy from a reactive to a proactive one, focusing on health management rather than disease treatment, is a major factor in these cost savings in case of cognitive impairments like Alzheimer Disease. AI-based technology will play a major role in helping individuals maintain their health through continuous monitoring and coaching and will ensure earlier diagnosis, treatments, and follow-ups.

In this paper, we investigate the use of blockchain-based deep neural networks for higher speed and delivery of healthcare data in a healthcare management system. The study exhibits a real-time health monitoring for classification and assesses the response time and accuracy.

The main contribution of the work involves the following:

- The authors investigate the use of blockchain-based deep neural networks for higher speed and delivery of healthcare data in a healthcare management system
- The authors develop a real-time health monitoring for classification and assess the response time and accuracy
- The authors analyse various classes to predict the brain disease as benign or malignant that includes AD, mild cognitive impairment, and normal cognitive level
- The authors develop a framework with a series of processing where most of the data are utilized for training these classifiers and ensemble model with a metaclassifier classifying the resultant class

## 2. Related Works

Distributed AI can be used to overcome the scalability, cost, and storage concerns of EHR among distributed nodes in the blockchain [11]. Similar to older classical machine learning (ML) and statistical methods [12], they employed raw data to choose appropriate characteristics and construct patterns of interest, rather than analysing the data itself. Deep learning (DL) approaches learn about feature selection from the data itself and then without any human intervention enable the discovery of hidden complex correlations within the data [13].

The article "Blockchain-Based Deep Learning to Process IoT Data Acquisition in Cognitive Data" was retracted in 2023. Reasons: signs of a paper mill; compromised peer review; unreliable results or conclusions.

Many academics have come up with effective ways to deal with the security and privacy problems of putting EHRs on blockchain. According to Esposito et al. [14], the patient privacy issues can be addressed by using blockchain technology to store EHR records. They did not discuss the internal structure and format of EHRs.

Logic expressions given by Chen et al. [15] were used to calculate EHR indices, which were then transferred to the blockchain network. As the number of transactions on the blockchain grows, the amount of overhead associated with index searching also grows, making it less scalable. An architecture devised by Amin et al. [16] for a single server that allows anonymity and resilience at lower communication costs was developed. There was no discussion of the trust difficulties that arise from long-term customer relationships.

An IoT-based RFID tag structure that is secure and anonymous at low latency was developed by Gope et al. [17] to combat impersonation attempts. In the current approach, the server identity can be hacked. FHIRChain, a healthcare blockchain developed by Zhang et al. [18], enables the identification of medical records and the authorization of access to them. But semantic interoperability is not addressed. For EHR data, feature selection and extraction of patient clinical data are also being done using DL frameworks.

A collaborative, distributed, federated deep learning model training for fairness and scalability on blockchain was proposed by Weng et al. [19]. For retrained models, however, the transfer learning function needs to be explored more thoroughly. Modeling time, admission procedures, and appropriate patient diagnosis were all accomplished using LSTM cells by Pham et al. [20].

By pretraining the word model word2vec, the authors of [21] used word embedding methodologies to tackle the hefty dictionary of 197,100 distinct medical abbreviations. Suo et al. [22] developed a convolutional neural network (CNN) that uses software cross-entropy loss to identify patient groups. Alhussein and Muhammad [23] used the transfer learning technique, which included the use of VGG-16 and Caffee. For clinical notes, Jacobson and Dalianis [24] used the word2vec-based embedding approach to compare stacked AEs and restricted Boltzmann machine (RBM).

EHR deployment in Healthcare 4.0 applications is a topic covered in the aforementioned debates. There have also been discussions on the security concerns of installing EHR on the blockchain and offered solutions including privacy-preserving ones [14], authentication and authorization utilising lattices [15], and lattices [25]. They did not solve the issue of transaction scalability. There have also been models based on feature parameters, pretrained models, and vector similarity [22, 24]. Security and prediction models work together in Healthcare 4.0 applications.

The article "Blockchain-Based Deep Learning to Process IoT Data Acquisition in Cognitive Data" was retracted in 2023. Reasons: signs of a paper mill; compromised peer review; unreliable results or conclusions.

As a result, this study provides a revolutionary architecture for Healthcare 4.0 applications that incorporates lattices, blockchains, and deep learning algorithms. For this study, the main goal is twofold. In mined transactions, the blockchain guarantees immutability and chronology. In addition, by using DNN prediction on previously recorded EHR feature records, it is possible to classify and display categorised findings to users more quickly. By automating recommendations, it cuts down on feature extraction time and boosts the scalability of mined transactions. Based on previous diagnoses and current health circumstances, suggestions are made. By averting serious sickness, it allows patients to receive treatment and medication on time, potentially saving their lives.

## 3. Proposed Method

In this, we use a blockchain network for faster transaction of data from the seed node to destination node with proper security. The sparse autoencoder is used for prediction of disease from the input collected datasets from IoT devices.  Figure 1 shows the process of data collection and processing using an effective blockchain and deep learning mechanism to identify the disease. It initially involves the collection of data, and then, the collected data is transmitted securely via blockchains. The stored data at the cloud servers are preprocessed, feature extracted, and then classified to identify the disease type.

### 3.1. Prediction Using a Sparse Autoencoder

As shown in Figure 1, an autoencoder network with a hidden layer may be used to learn certain compact characteristics from the data *x* = {*x*_1_, *x*_2_, *x*_3_, *x*_4_, *x*_5_} shown in Figure 2. Layer 1 represents the input layer, layer 2 represents the concealed layer, and layer 3 represents the reconstitution layer for the output layer. Reconstitution layer error is reduced as much as feasible as an aim of the training technique. The hidden layer might be considered a new sort of data representation because the data features can be retrieved from it.

To put it another way, the autoencoder network *h*_*W*,*b*_(*x*) ≈ *x* is to learn a given task. This arrangement has the ability to mine data for hidden features that are not readily obvious by restricting the number of neurons in the hidden layer. A 32 × 32 image can be processed by ten thousand twenty-four neurons, for example. Using an autoencoding network with a hidden layer of 50 neurons, it is possible to produce a compact representation of the image. In this way, PCA and dimension reduction methods perform the same function as they do in practise. However, the number of neurons in the buried layer is very low. It is possible to uncover underlying features even if the number of neurons in the hidden layer is large. A limitation on the network can lead it to become sparse if the activation value of each neuron in the hidden layer is optimized. If the input neurons are utilised, then the output neurons are also utilised.

(1) $$\begin{array}{c} \rho_{j}=\frac{1}{m}\overset{m}{\underset{i=1}{\sum }}a_{j}x_{i}, \end{array}$$

where *m* is the input neurons and *ρ*_*j*_ is the sparse parameter (0.05).

The article "Blockchain-Based Deep Learning to Process IoT Data Acquisition in Cognitive Data" was retracted in 2023. Reasons: signs of a paper mill; compromised peer review; unreliable results or conclusions.

The KL distance formulation is used to optimize the sparse parameter while solving the hidden layer.

(2) $$\begin{array}{c} \text{KL}\left(\rho \left\|\rho_{j}\right.\right)=\rho \log\frac{\rho }{\rho_{j}}+\left(1-\rho \right)\log\frac{1-\rho }{1-\rho_{j}}. \end{array}$$

In the convolution layer, the spatiotemporal convolution kernel simply gives the input of each feature map. When a network is configured manually, it has a limited ability to learn from its own experience and extract the most relevant aspects from the data. As illustrated in Figure 1, DNN uses a sparse autocombination technique that can automatically learn the combination of input feature maps that should be utilised as the input of the convolution layer.

The output of the neural network sparse autoencoder is subjected to the network sparse constraint. In this example, the input is constrained by the sparse constraint. These two forms of operation are different, but they accomplish the same things. Useful in a variety of industries and applications, the sparse autoencoder neural network extracts low-level properties from the input data. The output layer of the network is activated by using sparse limitations on the network output side. Accordingly, we will only activate neurons in the output layer that have been trained to respond to certain inputs in order to construct the most compact representation of input data—in other words, extract the most compact representation of data.

It is important to note that the previous layer input feature maps are used as inputs for each of the output feature maps in this framework spatiotemporal convolution. However, the number of feature maps that may be input into the output feature map is highly constrained because of the sparse restrictions.

## 4. Results and Discussions

In this section, we present the results of the proposed DNN-BC model and the existing smart contract with DNN, distributed blockchain with DNN, and multifactor authentication with DNN classification.

The article "Blockchain-Based Deep Learning to Process IoT Data Acquisition in Cognitive Data" was retracted in 2023. Reasons: signs of a paper mill; compromised peer review; unreliable results or conclusions.

The results are compared in terms of different performance metrics that include packet delivery rate, throughput, delay, and energy efficiency. It is further tested in terms of classification accuracy and loss. The simulation is conducted in Python3.8, where the CNN is modelled in TensorFlow2.2. The simulations are conducted on a high-end computing engine with 16 cores and 32 threads CPU, 16 GB of primary memory, and a graphics acceleration unit: GTX 1060. The simulation is conducted on a high-end computing platform that supports the implementation of blockchains and healthcare management system with a classification module.

Figure 3 shows the results of the packet delivery rate between the proposed DNN-BC model and the existing smart contract with DNN, distributed blockchain with DNN, and multifactor authentication with DNN classification. The results of simulation show that the proposed DNN-BC model has a higher rate of PDR in transmitting the data from a source to destination via blockchains.

Figure 4 shows the results of throughput between the proposed DNN-BC model and the existing smart contract with DNN, distributed blockchain with DNN, and multifactor authentication with DNN classification. The results of simulation show that the proposed DNN-BC model has a higher rate of throughput in transmitting the data from a source to destination via blockchains.

Figure 5 shows the results of delay between the proposed DNN-BC model and the existing smart contract with DNN, distributed blockchain with DNN, and multifactor authentication with DNN classification. The results of simulation show that the proposed DNN-BC model has reduced delay in transmitting the data from a source to destination via blockchains.

Figure 6 shows the results of energy efficiency between the proposed DNN-BC model and the existing smart contract with DNN, distributed blockchain with DNN, and multifactor authentication with DNN classification. The results of simulation show that the proposed DNN-BC model has increased energy efficiency in blocks while transmitting the data from a source to destination via blockchains.

The simulation is conducted to test the efficacy of the model over that of the OASIS-3 dataset, which is a longitudinal neuroimaging, cognitive, clinical, and biomarker dataset for normal aging and AD, and it is further trained and tested on the UDS dataset from ADNI.

Table 1 shows the results of classification accuracy between the proposed DNN-BC model and the existing smart contract with DNN, distributed blockchain with DNN, and multifactor authentication with DNN classification. The results of simulation show that the proposed DNN-BC model has increased classification accuracy in classifying the data instances in the healthcare field.

The article "Blockchain-Based Deep Learning to Process IoT Data Acquisition in Cognitive Data" was retracted in 2023. Reasons: signs of a paper mill; compromised peer review; unreliable results or conclusions.

Table 2 shows the results of classification loss between the proposed DNN-BC model and the existing smart contract with DNN, distributed blockchain with DNN, and multifactor authentication with DNN classification. The results of simulation show that the proposed DNN-BC model has reduced classification loss in classifying the data instances in the healthcare field.

## 5. Conclusions

In this paper, the study uses blockchain modelling-based DNN for optimal transmission of captured data from the sensing IoT node to the destination based on the user query. The study offers higher speed and delivery of data using a healthcare management framework. The testing on real-time data shows that the health monitoring and its classification provide increased accuracy with optimal response time based on the user query. The results of simulation show that the proposed method accurately responds to the query with high speed retrieval of classified results compared to other existing blockchain data transfer mechanisms. In future, the modelling of blockchain in a distributed ledger can be improvised with the utilization of machine learning or deep learning optimization that could be aimed at bringing effective ledgering of the addresses.

## Figures and Tables

**Figure 1:** Architecture diagram.

**Figure 2:** Sparse autoencoder.

**Figure 3:** Packet delivery rate (no unit).

**Figure 4:** Throughput (Mbps).

**Figure 5:** Delay (ms).

**Figure 6:** Energy efficiency (%).

**Table 1:** Classification accuracy.

Methods	Train accuracy	Test accuracy
Proposed DNN-BC	0.539	0.559
Multifactor authentication with DNN	0.553	0.524
Distributed blockchain with DNN	0.185	0.208
Smart contract with DNN	0.157	0.256

**Table 2:** Loss.

Methods	Train loss	Test loss
Smart contract with DNN	0.219	0.209
Distributed blockchain with DNN	0.212	0.227
Multifactor authentication with DNN	0.157	0.157
Proposed DNN-BC	0.156	0.210

## Data Availability

The datasets used and/or analyzed during the current study are available from the corresponding author on reasonable request.
